# Effects of miR-363 on the Biological Activities of Eutopic Endometrial Stromal Cells in Endometriosis

This article has been retracted.

**DOI:** 10.1155/2022/7663379

**Published:** 2022-03-26

**Authors:** Manman Nai, Yingying Zhang, Lei Li, Yuxi Jin, Yangge Li, Luwen Wang, Chenchen Ren

**Affiliations:** Department of Gynecology and Obstetrics, The Third Affiliated Hospital of Zhengzhou University, Zhengzhou, 450052 Henan Province, China

## Abstract

EMs is a kind of benign disease with certain malignant behaviors. The adhesion, invasive growth, and angiogenesis of ectopic endometrial cells are the pathological basis of EMs occurrence, but its etiology and pathogenesis have not been completely illustrated yet. In our research, we aim to investigate the role of miR-363 in the pathogenesis of endometriosis. Real-time quantitative PCR was used to detect the expression of miR-363 before and after ESC/NSC transfection. CCK-8, flow cytometry, and transwell assay were used to detect the effect of the miR-363 expression on cell proliferation, apoptosis, and invasion. The effects of the miR-363 expression on the contents of Fas/APO-1 and ICAM-1 in cell culture supernatant were detected by ELISA. qRT-PCR and WB assay were used to detect the effects of the miR-363 expression on the mRNA and protein expression levels of ICAM-1, MMP-7, and VEGF in ESC. The increased expression of miR-363 could inhibit the proliferation and invasion of ESC, promote apoptosis, and inhibit the secretion of FAS/APO-1 and ICAM-1. The knockdown expression of miR-363 promoted proliferation and invasion of NSC, inhibited apoptosis, and promoted secretion of FAS/APO-1 and ICAM-1. VCAM-1, VEGF, and MMP-7 were detected in ESCs before transfection. The protein expression level was higher than that of NSCs. Compared with pretransfection, the protein levels of VCAM-1, VEGF, and MMP-7 in the M-363 group were significantly downregulated. The downregulated expression of miR-363 was associated with a stronger cell proliferation ability, a lower cell apoptosis rate, and a stronger ESC. Migration is associated with invasiveness, proliferation, angiogenesis, and immune escape. The low expression of miR-363 promotes endogenesis through posttranscriptional regulation of target genes VCAM-1, MMP-7, and VEGF. The differential expression of miR-363 between ESC and NSC may be an important factor in the many biological differences between ESC and NSC.

## 1. Introduction

Endometriosis (EMs) is a common gynecological endocrine disease, which is characterized by the extrauterine proliferation and invasive growth of endometrial cells [1]. EMs shows malignant biological behaviors, where the epithelial and mesenchymal cells on the abnormal endometrium can migrate and adhere to and invade the ovary, peritoneum and rectum [2]. The pathogenesis of EMs remains unclear at present, and none of the existing theories can completely explain the causes of EMs pathogenesis. The pathogenesis of EMs involves multiple factors; for instance, hormone environment, genetic predisposition, immunologic derangement, and environmental factors can promote the genesis of EMs [3–5]. In addition, it is suggested by the “eutopic endometrium determinism” that the special biological characteristics of EM eutopic endometrium, such as stronger ectopic implantation, invasion, and angiogenesis, are related to its pathogenesis [6]. This may be derived from the abnormal gene expression, but the precise mechanism remains incompletely illustrated yet.

As a naturally formed posttranscriptional regulatory factor, miRNAs are the regulatory factors that regulate gene expression at posttranscription level; besides, miRNAs have a series of extensive target mRNAs, and over 50% miRNAs are located in tumor-related genomic domains and fragile sites [7], implying that the disordered miRNA expression will exert a vital role in the pathogenesis of proliferative disease. Therefore, changing miRNA expression can lead to abnormal expression of many genes and gene products, thus significantly affecting cell viability. Consequently, research on the expression and roles of miRNAs in diseases like tumor has become a persistent hotspot. As a result, the differential miRNA expression profiles among EMs patients may be the important cause of its pathogenesis [8], finally controlling the disease occurrence. MicroRNA-363 (miR-363) is one of the miRNAs screened to be downregulated in papillary thyroid cancer [9]. Previous experiments prove that the miR-363 overexpression inhibited the invasion ability of endometrial stromal cells [10], proving that the abnormal expression of miR-363 may be of important significance in the pathogenesis of EMs. Some research verifies that the miR-363 expression is downregulated in multiple malignant tumors, which significantly promotes tumor cell growth and proliferation [11–13]. In addition, bioinformatic analysis results suggest that VCAM-1, MMP-7, and VEGFA are the predicted target genes of miR-363: VCAM-1 plays a characteristic role in vascular endothelial cell and immune cell adhesion[14].

Fas (Apo.1 or TNFRSF6) is a type I transmembrane glycoprotein with the molecular weight of 45 kDa, which belongs to the TNF nerve growth factor receptor family. The Fas/FasL system plays crucial roles in physiological homeostasis and pathological status, including cell escape of immune surveillance. MMP-7 can degrade the extracellular matrix (ECM) in the physiological and pathological processes[15][14], and vascular endothelial growth factor (VEGFA) is an important angiogenesis mediator[15]. As is known to all, the enhanced cell adhesion, migration, invasion, and angiogenesis are the important pathological basis of EM pathogenesis. The biological behaviors of endometrial tissues in EMs are similar to tumor growth, which is related to the changed biological characteristics. Thus, it is speculated that miR-363 may play a crucial role in the pathogenesis of EMs. At present, reports regarding the role of miR-363 in EM genesis and development are lacking. This experiment changed the miR-363 expression in endometrial stromal cells (ESCs), detected its effect on the biological behaviors of endometrial cells, verified the targeted regulatory relationship of miR-363 with the genes related to the EM pathogenesis, and explored the value of miR-363 in EM pathogenesis.

## 2. Materials and Methods

### 2.1. Subjects

All the 30 cases who were diagnosed with EMs at the Gynecology and Obstetrics and received total hysterectomy from January to December 2019 were enrolled as the experiment group. At the same time, 30 cases with cervical intraepithelial neoplasia (CIN) who received total hysterectomy were enrolled as the control group. The average age in the experiment group was (43.19 ± 0.74) years, while that in the control group was (41.04 ± 0.82) years, and there was no statistical difference between the two groups (*P* = 0.55). All patients had regular menstruation, with no other surgical, endocrine, immune, or metabolic disease; besides, they did not receive GnRH analogue, hormone drug, and antibiotic treatment within three months before surgery. The eutopic endometrium at late secretion stage (verified by the menstrual cycle and histological examination) was scraped under sterile condition immediately after the surgery, followed by immediate cell culture. The specimen collection protocol was approved by the Ethics Committee of the hospital, and all patients had signed the informed consent. The diagnosis of all cases was verified through postoperative pathology.

### 2.2. Isolation, Primary Culture, and Identification of ESCs

The endometrial tissues were washed with PBS thrice to remove the blood stains, cut into pieces (1 mm [3] or smaller, paste under naked eyes) with the ophthalmic scissors into the small beaker, and digested with 10 volumes of type I collagenase (final concentration, 1 mg/ml). After repeated blowing, the endometrial tissues were transferred into the centrifuge tube to incubate for 1 h at 37°C in the incubator, and the centrifuge tube was vibrated once every 15-20 min, so that the samples were sufficiently contacted and digested. After the tissues became flocculent, they were filtered with the 200-mesh sieve, and the filtrate was collected and added into the centrifuge tube for 5 min of centrifugation at 800 rpm. After discarding the supernatant, cells were resuspended with DMEM/F-12 cell culture medium containing 10% FBS, filtered with the 400-mesh sieve, and the filtrate was cultured in the cell culture box under 37°C and 5% CO_2_ conditions. The cell culture medium was replaced at 24 h later. Thereafter, cells were inoculated into the 48-well plate at 1 × 10^6^/ml and were identified after achieving 70-80% confluence. Then, cells were fixed with 4% paraformaldehyde (PFA) for 4 min at 4°C; after adding the RIPA lysate, the cells were allowed for 20 min of standing at room temperature in accordance with the biotin-SPTM immunohistochemical assay kit instructions, with the working concentrations of primary antibodies (vimentin and keratin antibodies) being 1 : 200. Cells whose cytoplasm was brown were deemed as the positive cells.

### 2.3. Targeted Change of the miR-363 Expression

The experiments with in situ endometrial mesenchymal cells were divided into three groups. The groups were transfected with miR-363 mimics (ESC-m363), transfected with negative control (ESC-NC), and transfected with miR-363 inhibitors (ESC-in363). Transfection was performed using the Lipofectamine 2000 transfection reagent. Stromal cells of normal endometria in endometriosis patients (NSCs) were divided into three groups: the miR-363 inhibitor group (NSC-in363 group, containing miR-363 inhibitors, lipofectamine 2000-containing), negative control (NSC-NC group, inhibitor negative control, lipofectamine 2000-containing), and blank group (NSC-Blank group, no small fragment RNA, no lipofectamine 2000). Each group contained 20 samples. It is currently known that miRNAs bind with the complementary sequences in the 3′UTR of target genes regulate the target gene expression through directly degrading mRNA or suppressing protein synthesis, control growth, development, proliferation, apoptosis, and stress response through modulating the gene expression. The 2-8 most important bases at the identifiable binding sites on the miRNA sequence are referred to as “seed region.” It was verified experimentally that, in ESCs, miR-363 bounds to the 3′UTR of the predicted target genes VCAM-1, MMP-7, and VEGFA through the seed region; in addition, the protein levels of three groups of genes were suppressed by miR-363 mimics and upregulated by miR-363 inhibitors, while the mRNA expression levels exhibited no changes. These results pointed out that miR-363 specifically regulated the expression of VCAM-1, MMP-7, and VEGFA at posttranscriptional level.

### 2.4. miR-363 Expression Detected by Real-Time Fluorescent Quantitative PCR

The total cellular RNA was extracted by the TRIzol method, which was then prepared into cDNA in accordance with the reverse transcription kit instructions. Then, the gene fragments were amplified. The miR-363 and stem-loop internal reference U6 primers were obtained from RiboBio Co., Ltd. The reaction conditions were as follows: the initial denaturation conditions were basically consistent with denaturation conditions for every gene, as shown below: initial denaturation at 95°C for 30 s, followed by 40 cycles at 95°C for 40 s and 60°C for 5 s. The 2^-*ΔΔ*Ct^ method was adopted to calculate the relative expression level of the target gene.

### 2.5. Cell Proliferation Assay

Cells from each group were inoculated into the 96-well plates, the medium was replaced at 24 h later, 5 wells were prepared for each group, and the transfected cells were grouped as mentioned above. At 48 h later, the medium was replaced, CCK-8 solution was added, and the absorbance (*A*) value was measured with the microplate reader. The assay was repeated thrice, and the average was taken.

### 2.6. Cell Apoptosis Detected by Flow Cytometer

Cells in each group were transfected for 48 h and digested with EDTA-free trypsin. Then, cells were washed with PBS twice and collected (1 ~ 5 × 10^5^) by 5 min of centrifugation at 2000 rpm. Later, 500 *μ*l Binding Buffer was added to suspend cells; after the addition of 5 *μ*l Annexin V-FITC, 5 *μ*l propidiumlodide was added and mixed sufficiently, followed by reaction for 5-15 min in dark at room temperature. Flow cytometry was conducted within 1 h.

### 2.7. Transwell Invasion Assay

[9, 10]. The Matrigel was thawed at 4°C and diluted with serum-free DMEM at a ratio of 1 : 8; then, the mixed solution was added into the upper Transwell chamber at 60 *μ*l medium/well to incubate for 4 h under 37°C and 5% CO_2_ conditions. Then, the cells were starved with the serum-free DMEM for 24 h, prepared into single-cell suspension with DMEM containing 15% fetal bovine serum (FBS), and 200 *μ*L cell suspension was collected and inoculated into the upper chamber at 1 × 10^5^/well as the blank control. Six duplicate wells were set for each group (*n* = 4 groups), and altogether, 24 wells were set. Cells were later cultured for 48 h under 37°C and 5% CO_2_ conditions. Afterwards, the Transwell chambers were taken out and washed with PBS twice, cells on the upper chamber surface were wiped off with the cotton ball, while cells on the lower chamber surface were fixed with 95% ethanol for 10 min and stained with hematoxylin and eosin (HE), and then the number of cells invading the lower chamber surface was counted under the microscope. Cells in five fields of view (FOVs, ×400) were counted randomly to take the average. The invasion inhibition rate is as follows: (%) = (1 − invading cell number in experiment group/invading cell number in control group) × 100%. Fas/apo-1 and ICAM-1 contents in the cell culture supernatant were detected by enzyme-linked immunosorbent assay (ELISA). The supernatant was collected for detection in accordance with the ELISA kit instructions.

### 2.8. Construction of MMP-7, VEGF, and VCAM-1 Vectors and Luciferase Activity Analysis

The VCAM-1, MMP-7, and VEGF luciferase reporter plasmids were constructed by Shanghai GEMMA. It is necessary to construct a new blood supply for the survival of ectopic endometrium and the development of EMs. Vascular endothelial growth factor (VEGF) is an important angiogenesis mediator and a potent inducer to promote endothelial cell division, morphogenesis, and vascular permeability. Some research suggests that VEGF is highly expressed in EMs and activated by macrophages. Also, it is found that the VEGF levels significantly increase in the ectopic lesions and peritoneal fluid of EMs patients, and the increased VEGF can promote new vessel formation and enhance the interaction between endometrial cells and the surrounding tissues and environment. This study indicated that the downregulated miR-363 promoted the VEGF expression. These results support the previous research results and reveal that the stronger new vessel formation ability in EMs can be controlled by regulating the miR-363 expression.

After construction, the VCAM-1/MMP-7/VEGFA luciferase reporter plasmids were cotransfected with miR-363 mimics and Prl-TK Renilla luciferase plasmid into ESCs using the lipofectamine 2000 kit. The grouping is shown below in Table 1. The Firefly and Renilla luciferase activities were detected continuously at 48 h after transfection using the Dual-Glo ® Luciferase Assay System kit.

### 2.9. Expression of VCAM-1, MMP-7, and VEGF Proteins Detected by Western Blotting

The total cellular proteins were collected for SDS-polyacrylamide gel electrophoresis; after membrane transfer, primary antibody solution (1 : 400 for primary antibody, 1 : 2000 for GAPDH, diluted with the blocking buffer) was added and incubated overnight at 4°C on the shaking table. Afterwards, a secondary antibody was added to further incubate the proteins, followed by chemiluminescence, developing, and fixing. Gray level was analyzed using the Quantity One software, and the gray level ratio of the target band to GAPDH was treated as the relative expression quantity of the target protein.

## 3. Statistical Analysis

Data were analyzed using the SPSS18.0 software, and the reference ranges of data were expressed as mean ± standard error. For normally distributed data, the *t*-test was adopted for the comparison of means between two groups, while *F*-test was applied for comparison among multiple groups. For data conforming to homogeneity of variance, Tukey test was adopted for multiple comparisons of means among several groups, while for data not conforming to heterogeneity of variance, Games-Howell test was employed for multiple comparisons of means among several groups. A difference of *P* < 0.05 indicated statistical significance.

## 4. Results

### 4.1. Cell Identification

Cells cultured to the third passage were identified through immunohistochemistry (IHC). As shown in Figure 1, vimentin and CD10 staining showed a positive reaction (Figures 1(a) and 1(c)), verifying that the cells adopted in this experiment were ESCs. In addition, cytokeratin, VIII factor, and leukocyte common antigen (LCA) (Figures 1(b), 1(d), and 1(e)) showed a negative reaction, proving that the cultured cells were not mixed with epithelial cells, endothelial cells, or white blood cells. As shown in Figure 1, Vimentin and CD10 (Figures 1(a) and 1(c)) showed positive reaction, whereas cytokeratin, VIII factor, and LCA (Figures 1(b), 1(d), and 1(e)) showed negative reaction.

### 4.2. Effects of Transfection with miR-363 Mimics/Inhibitors on the miR-363 Expression Level

As shown in Figure 2(a), ESCs transfected with the FAM-labeled miR-363 mimics were observed under the fluorescence microscope, which revealed that the small RNA fragments were transfected into cells. It was illustrated by the real-time PCR results from Figure 2(b) that, when the relative miR-363 expression level of one random NSC was regarded as 1, the relative miR-363 expression level (2974.21 ± 368.82) in ESCs after miR-363 mimics transfection showed significant difference compared with that before transfection. The miR-363 expression in ESCs transfected with NC (0.52 ± 0.16) and blank control (0.55 ± 0.14) displayed no obvious change (*P* = 0.924). After transfection with miR-363 inhibitors, the relative miR-363 expression level in NSCs (0.08 ± 0.01) was significantly downregulated compared with that before transfection (*P* = 0.001), while those in NSCs transfected with iNC (0.84 ± 0.11) and blank control (0.82 ± 0.05) showed no obvious change (*P* = 0.826).

### 4.3. Effects of miR-363 Expression on the ESC Proliferation and Apoptosis

It was shown in Figure 3(a) that, before transfection, ESCs showed a higher proliferation rate than NSCs (*P* < 0.05). Compared with that before transfection, the proliferation rate of the miR-363 group significantly decreased at 24, 30, 36, and 48 h (*P* < 0.05 at all time points), and the growth curve almost coincided with that of NSCs, while the proliferation rate of NC group was not changed (*P* > 0.05 at all time points). The proliferation rate of the in-363 group at 24, 30, 36, and 48 h significantly increased (*P* < 0.05 at all time points), while that of the iNC group remained unchanged (*P* > 0.05 at all time points).

It was observed from Figure 3(b) that, before transfection, the ESCs apoptosis rate was lower than that of NSCs (*P* < 0.01). The apoptosis rate of the m-363 group was higher than those of the NC group and ESCs group (*P* < 0.01). The apoptosis rate of the in-363 group was lower than those of the iNC group and NSC group (*P* < 0.05). When comparing the NC group with the ESC group before transfection and the iNC group with the NSC group before transfection, the apoptosis rate exhibited no obvious change (NC vs. ESCs, *P* > 0.05; iNC vs. NSCs, *P* > 0.05).

### 4.4. Effects of miR-363 on ESC Invasion

As observed from Figure 4, before transfection, the number of cells penetrating the Matrigel in the ESC group was higher than that in the NSC group (*P* < 0.01). After transfection with miR-363 mimics, the number of cells penetrating the Matrigel in the m-ESC group was lower than that of the NC group and ESC group (*P* < 0.01). On the contrary, after transfection with miR-363 inhibitors, the number of cells penetrating the Matrigel in the in-363 group was higher than those of the iNC group and NSC group (*P* < 0.05). Compared with pretransfection, the numbers of cells penetrating the Matrigel in the iNC group and NSC group showed no obvious changes (NC vs. ESCs, *P* > 0.05; iNC vs. NSCs, *P* > 0.05).

### 4.5. Effects of the miR-363 Expression on the Adhesion and Immunocompetence of ESCs

As presented in Figure 5, before transfection, ESCs secreted higher levels of fas/apo-1 and ICAM-1 than NSCs. Compared with pretransfection, the increased miR-363 expression reduced the fas/apo-1 and ICAM-1 levels secreted by ESCs (*P* < 0.05 for two proteins); after transfection with NC, the levels of two proteins secreted by ESCs were not changed (*P* > 0.05 for two proteins). Meanwhile, decreasing miR-363 expression increased the fas/apo-1 and ICAM-1 levels secreted by NSCs (*P* < 0.05 for two proteins); after transfection with iNC, the two proteins secreted by NSCs showed no changes (*P* > 0.05 for two proteins).

### 4.6. miR-363 Specifically Regulated VCAM, VEGF, and MMP-7 in ESCs

VCAM-1 plays a characteristic role in the human immune system and is expressed in multiple cell types, including inflammatory cells and ESCs. VCAM-1 exerts a crucial part in inflammatory processes like white blood cell adhesion into blood vessel, endothelial migration, and white blood cell aggregation. It is pointed out that VCAM-1 changes with the menstrual cycle, verifying that VCAM participates in the physiological process of endometrium. As observed from Figure 6(a), after pMIR-VCAM-3′UTR, pMIR-MMP7-3′UTR, and pMIR-VEGF-3′UTR were transfected into miR-363, their luciferase activities were significantly lower than those in NC and blank control transfection groups (*P* < 0.05 for three groups of genes). There was no significant difference in the relative luciferase activity among these three in the NC or blank control transfection group (*P* > 0.05 for three groups of genes); moreover, there was no significant difference compared with the relative luciferase activity of pMIR-reporter (*P* > 0.05 for three groups of genes).

The expression of VCAM-1, VEGF, and MMP-7 before and after miR-363 transfection was analyzed by real-time PCR and Western blotting. Real-time PCR analysis indicated that, before transfection, the mRNA expression levels of VCAM-1, VEGF, and MMP-7 were upregulated in ESCs compared with NSCs (*P* < 0.001 for three groups of genes, Figure 6(b)); compared with pretransfection, the changes in the miR-363 expression did not affect the mRNA expression levels of VCAM-1, VEGF, and MMP-7 (m-363 vs. ESCs, in-m-363 vs. NSCs *P* > 0.05, Figure 6(b)). Western blotting results suggested that, before transfection, the protein expression levels of VCAM-1, VEGF, and MMP-7 were upregulated in ESCs compared with NSCs (*P* < 0.001 for three groups of proteins, Figure 6(c)). Compared with pretransfection, the protein expression levels of VCAM-1, VEGF, and MMP-7 in the m-363 group were significantly downregulated (*P* < 0.05 for three groups of proteins). In addition, the protein expression levels of VCAM-1, VEGF, and MMP-7 in the in-363 group were upregulated (*P* < 0.01 for three groups of proteins), while those in negative control groups (sNC and iNC groups) showed no obvious changes before and after transfection (sNC vs. ESCs *P* > 0.05, iNC vs. NSCs *P* > 0.05, Figures 6(c) and 6(d)). As speculated by our results, the low expression of miR-363 in ESCs might increase the MMP-7 translation to enhance the ESC invasion capacity. Invasion is of great importance to the genesis and development of EMs, which means the beginning of tissue remodeling on the basis of gene expression changes. The increased MMP-7 can enhance the invasion of surrounding tissues by the ectopic lesion; moreover, it is suggested in research that MMP-7 can stimulate endothelial cell growth, accelerate their migration, and participate in the occurrence of osteogenesis.

## 5. Discussion

miRNA can regulate the gene expression stability and exerts vital parts in multiple life activities, such as cell growth, differentiation, apoptosis, inflammation, and immune response [16]. According to estimates, about 30% of genes are regulated by miRNA. Therefore, the disordered miRNA expression may induce the abnormal expression of many related genes, leading to cell dysfunction. This implies that the disordered miRNA expression plays an important role in the pathogenesis of proliferative disease. miRNA regulates its extensive target genes to change the physiological and biological characteristics of endometrium [17]. miR-363 is located in chromosome X q26.2. This gene is involved in regulating multiple life activities, such as proliferation, invasion, and angiogenesis; besides, it is related to several malignant biological behaviors. However, the role of miR-363 in the pathogenesis of EMs remains unclear at present. This experiment points out that the changes in the miR-363 expression affected the biological functions of endometrial cells and regulated their malignant behaviors. The high level of sfas in peritoneal fluid of EMs patients and the high expression of fasL in immune cells will increase the fas-mediated immune cell apoptosis in the abdominal cavity, reduce the immune scavenging activity, and protect the ectopic endometrium, and all of these contribute to the survival of ectopic cells and the genesis and development of EMs. Thus, it can be speculated that miR-363 may regulate endometrial cell apoptosis through the fas/fasl pathway, protect the endometrial cells from programmed death, and finally promote EMs occurrence.

Under normal physiological status, cell proliferation and apoptosis are in a balance. The increased cell proliferation capacity and decreased apoptosis will lead to disordered cell viability. Moreover, the periodical change of endometrial cell apoptosis in EMs patients disappears; in particular, the endometrial cell apoptosis index significantly declines at the late secretion stage, which together with the persistent cell proliferation ability is the major cause of EMs occurrence [18, 19]. Endometrial cell invasion and penetration are the key factors related to the EMs pathogenesis. As suggested by our experimental results, the low expression of miR-363 promoted ESC invasion, while the high expression of miR-363 suppressed their invasion. The intercellular adhesion molecule-1 (ICAM-1) is a ligand of *β*2 integrin molecule, and its expression in inflammatory response and immune response has played an important role in the invasion and migration of lymphocytes and phagocytes to tissues; besides, it promotes the functions of antigen presenting cells [20]. This study discovered that the overexpression of miR-363 suppressed the secretion of ICAM-1, while downregulating the miR-363 expression increased its secretion. Some research suggests that the mRNA and protein expression of ICAM-1 increases in ESCs, and upregulating ICAM-1 promotes the adhesion capacity of ESCs. Noteworthily, sICAM-1 is mainly derived from ESCs. The serum ICAM-1 level is related to the sICAM-1 level and range secreted by endometrial cells, which is closely correlated with the disease severity. At present, it has been discovered that the origin and number of EMs lesions are directly related to the sICAM-1 content. Thus, it is speculated that the elevated sICAM-1 levels in abdominal and peritoneal cavities lead to the enhanced adhesion capacity of endometrial cells and promote the formation of ectopic lesion. Additionally, sICAM-1 can bind onto the NK cell surface, interfere with the NK cytotoxicity, and reduce the NK cells-mediated ectopic endometrial cell scavenging capacity, thereby leading to the occurrence of EMs [21, 22]. In mesenchymal stem cells (MSCs), the higher expression of ICAM-1 and VCAM-1 indicates the greater immunosuppression. This facilitates the endometrial cells to escape the effects of immunologic effector cells in the abdominal cavity. Therefore, it is speculated that the low expression of miR-363 can enhance the cell adhesion capacity and further protect the ectopic endometrial cells, thus further accelerating EMs occurrence. Consequently, in EMs, the downregulated miR-363 promotes the expression of VCAM-1, which may enhance the stimulation of inflammatory factors and promote cell (including vascular endothelial cells) adhesion at the inflammatory sites. In addition, in ectopic ESCs, ICAM-1 is regulated by the cytokine VCAM-1 in the abdominal cavity and exerts a role in the pathogenesis together with the latter. Some research suggests that the FasL mRNA expression increases in the activated peripheral blood mononuclear cells (PBMCs) and immune cells in the ectopic endometrial tissues. Cells expressing Fas can interact with FasL, inducing the programmed cell death [23]. The miR-363 expression is downregulated, which results in the increased level of soluble fas (sfas) in the extracellular environment, while sfas competitively antagonizes the combined fas and mitigates the apoptosis of endometrial cells.

The invasive characteristics of endometrium are related to the increased proteolysis activity. MMP-7 is also called the stromatolysis factor 1, which belongs to the MMP family highly expressed in tumor and has extensive substrate specificity. It can degrade extracellular matrix in the physiological and pathological processes and promote tumor cell invasion, development, and poor prognosis. It can be speculated based on our experimental results that, compared with the traditional hormone regulation-based treatments, upregulating the miR-363 expression can more effectively suppress the translation of EMs-related genes and downregulate the protein products associated with its execution function, which will effectively prevent the development of EMs. The strategy of regulating miRNA expression to control EMs development may serve as the treatment for EMs in the future.

## 6. Conclusion

To sum up, our research verifies that the downregulated miR-363 is related to the stronger invasion, apoptosis and proliferation, angiogenesis, and immune escape of endometrium, which provide further evidence for the role of miR-363 in the pathogenesis of EMs. It is speculated from this experiment that miR-363 regulates the gene expression products involved in the EM pathogenesis (such as VCAM, MMP-7, and VEGF) to regulate the eutopic and ectopic endometrial cell activity and affect the EMs pathogenesis. The differential expression of miR-363 between ESCs and NSCs is related to the biological differences between the two, which may be the key factor that participates in the EMs occurrence and development. However, there are still some shortcomings in our study. We need to conduct more detailed data analysis to achieve more scientific results.

## Figures and Tables

**Figure 1:** Third passage ESCs cultured in this experiment.

**Figure 2:** Changes in miR-363 expression level before and after transfection. (a) Cells transfected with FAM-labeled miR-363 mimics observed under the fluorescence microscope. A-1: FOV of ×100 magnification under the phase contrast microscope; A-2: FOV of ×100 magnification under the fluorescence microscope, where green fluorescence was observed in cytoplasm. (b) Changes in miR-363 expression level before and after transfection detected by real-time PCR. The results were expressed as mean ± standard error. B-1: The miR-363 expression level in ESCs elevated after miR-363 mimics transfection; B-2: The miR-363 expression level in NSCs decreased after miR-363 inhibitors transfection. M-miR-363: miR-363 mimics; in-miR-363: miR-363 inhibitors.

**Figure 3:** Effects of the miR-363 expression on the ESC proliferation and apoptosis. (a) Effects of changes in miR-363 expression on ESC proliferation detected by CCK-8 assay. (b) Effects of changes in the miR-363 expression on ESC apoptosis detected by flow cytometry.

**Figure 4:** Effects of miR-363 on ESC invasion detected through the Transwell invasion assay. (a) After transfection with miR-363 mimics, the cell invasion capacity declined, while after miR-363 inhibitor transfection, the cell invasion capacity increased. (b) The images showed the changes in ESC invasion capacity before transfection and after transfection with miR-363 mimics and NC and the changes in NSC invasion capacity before transfection and after transfection with miR-363 inhibitors and iNC.

**Figure 5:** Effects of the miR-363 expression on Sicam-1 (a) and sfas/apo-l (b) secreted by ESCs. Data were expressed as mean ± standard error. (a) Relative secretion levels of sICAM in the culture medium before and after transfection. (b) Relative secretion levels of sfas/apo-1 in the culture medium before and after transfection.

**Figure 6:** The relationship between VCAM-1, VEGF, MMP-7, and miR-363. (a) The direct binding relationships of miR-363 with VCAM-1, VEGF, and MMP-7 were verified through the dual-luciferase reporter system. (b) The mRNA expression levels of VCAM-1, VEGF, and MMP-7 after transfection with miR-363 mimics, miR-363 inhibitors, and corresponding negative controls were detected by real-time PCR. (c, d)The protein expression levels of VCAM-1, VEGF, and MMP-7 after transfection with miR-363 mimics, miR-363 inhibitors, and corresponding negative controls were detected by Western blotting. GAPDH was used as the internal reference.

**Table 1:** Grouping of dual-luciferase reporter gene system.

Group intervention factor	Eutopic ESCs					
pMIR-REPORT™	+	+	-	-	-	-
pMIR-VCAM1-3′UTR/	-	-	+	+	-	-
pMIR-MMP7-3′UTR/						
pMIR-VEGF-3′UTR						
miR-363 mimics	+	-	+	-	+	+
Negative control	-	+	-	+	-	-

Notes: “+” indicates that the factor is added, while “-” suggests that the factor is not added.

## Data Availability

The datasets used and/or analyzed during the current study are available from the corresponding author on reasonable request.
